# Unbalanced Fault Diagnosis Based on an Invariant Temporal-Spatial Attention Fusion Network

**DOI:** 10.1155/2022/1875011

**Published:** 2022-03-30

**Authors:** Jianhua Liu, Haonan Yang, Jing He, Zhenwen Sheng, Shou Chen

**Affiliations:** ^1^College of Railway Transportation, Hunan University of Technology, Zhuzhou 412007, China; ^2^College of Electrical and Information Engineering, Hunan University of Technology, Zhuzhou 412007, China; ^3^Shandong Xiehe University, Jinan 250000, China; ^4^Shenzhen Beauty Star Co., Ltd., Shenzhen 518000, China

## Abstract

The health status of mechanical bearings concerns the safety of equipment usage. Therefore, it is of crucial importance to monitor mechanical bearings. Currently, deep learning is the mainstream approach for this task. However, in practical situations, the majority of fault samples have the issue of severe class unbalancing, which renders conventional deep learning inapplicable. Targeted at this issue, this paper proposes an invariant temporal-spatial attention fusion network called ITSA-FN for bearing fault diagnosis under unbalanced conditions. First, the proposed method utilizes the invariant temporal-spatial attention representation section, which consists of a pretrained convolutional auto-encoder model, a convolutional block attention module, and a long short-term memory network, to extract independent features and invariant features of spatial-temporal characteristics from input signals. Then, a multilayer perceptron is used to fuse and infer from the extracted features and design a new loss function from the focal loss for network training. Finally, this article validates proposed model's effectiveness through comparative experiments, ablation studies, and generalization performance experiments.

## 1. Introduction

Rolling bearings play a key role in mechanical equipment. Any tiny fault can affect the operation of the equipment or even produce latent threats to lives and property [1–4]. Therefore, it is necessary to monitor the health status of mechanical equipment. In recent years, deep learning has been used widely in the field of intelligent fault diagnosis of machinery [5–8]. Wang et al. proposed a deep learning similarity measure model for machine status classification [9]. Zheng et al. combined a capsule neural network and an abnormal module (XCN) and applied them to intelligent fault diagnosis [10]. Li et al. proposed a self-adaptive method in the field of mechanical fault diagnosis based on deep learning [11]. The abovementioned works have achieved good results in certain scenarios. However, these methods are mostly based on balanced mechanical datasets and disregard the situation of unbalanced mechanical statuses. In reality, normal equipment samples are usually redundant, whereas the instances of faulty samples are rare. This unbalanced sample distribution renders conventional deep learning prone to biased attention (i.e., learning class features more from large populations while disregarding features of small populations), resulting in deteriorated identification accuracy.

Targeting the unbalanced data issue in fault diagnosis, researchers have proposed a variety of methods [12–14]. Currently, solutions to unbalanced classification mainly fall into two categories: data-level methods and algorithm-level methods. Data-level methods include oversampling for small population classes and undersampling for large population classes. State-of-the-art research favors the former [15]. Regarding the oversampling method, random oversampling (RAMO) is the simplest oversampling technique, but it is prone to overfitting [16]. Therefore, Chawla et al. proposed a synthetic minority oversampling technique (SMOTE) to solve this problem by interpolating new synthetic samples [17]. However, SMOTE has the issues of overgeneralization and noise sensitivity. To address this issue, Bunk et al. proposed the Safe-level-SMOTE technology, which uses the K-nearest neighbor sample distribution to determine the “safety level” value and then synthesizes a new instance close to the maximum safety level [18]. Although Safe-level-SMOTE has certain advantages over SMOTE, its new instance usually has the problem of being far away from the decision boundary. In addition, Borderline-SMOTE (BSMOTE) [19], Cluster-SMOTE [20], Adaptive Synthetic Sampling (ADASYN) [21], Kmeans-SMOTE [22], and other cluster sampling methods are also achieved good results. However, these methods all rely excessively on the value of the parameter *k*. Thus, some weighting methods that do not rely on the nearest-neighbor method to obtain boundary instances are proposed, for example, majority weighted minority oversampling technology (MWMOTE), cluster-based majority weighted minority oversampling (Cluster-MWMOTE) [23], sample feature oversampling (SCOTE) [24], and expectation maximization local weighting minority oversampling (EM-LWMOTE) [25]. In addition to the abovementioned oversampling methods, deep generator models have also been widely used in the field. Li et al. proposed the assistant classifier Wasserstein generative adversarial network with gradient penalties (ACWGAN-GP) to generate high-quality samples for the minority class [26]. Yang et al. solved the unbalanced data issue through a data generation method based on a generative adversarial network and then utilized the multiscale convolutional neural network (MSCNN) for fault diagnosis on a harmonic drive [27]. Wang et al. designed the conditional variation auto-encoder generative adversarial network (CVAE-GAN) for unbalanced fault diagnosis [28]. The abovementioned methods achieved good results. However, on one hand, these methods may miss latent valuable information and, on the other hand, may produce additional computation loads to the networks. Therefore, for practical industrial cases, oversampling methods are usually not a good solution.

For algorithm-level methods, cost-sensitive learning is the mainstream way to deal with imbalanced classification problems [15]. It is a learning paradigm that allocates the cost of misclassification to the categories involved in the classification task. Existing cases include cost-sensitive neural networks [29], cost-sensitive decision trees [30], and cost-sensitive extreme learning machines [31]. However, most of these cases belong to the category of machine learning, and there are relatively few studies on deep neural networks. Thus, Peng et al. proposed a new type of bidirectional gated recurrent unit (BGRU) and combined it with a cost-sensitive active learning strategy for fault diagnosis [32]. Zhang et al. proposed the evolutional cost-sensitive deep belief network (ECS-DBN) for unbalanced classification in which misclassification costs on training dataset are optimized through self-adaptive differential evolution [33]. In addition, in terms of cost-sensitive online learning, based on the cost-sensitive learning framework [34], cost-sensitive online gradient descent (COG) was proposed. However, COG was limited to only extracting first-order information of the sample (weighted average of the gradient). To solve this problem, Zhao et al. proposed a series of cost-sensitive online classification algorithms with self-adaptive normalization and validated them [35]. It is worth mentioning that the key to these methods is to determine the cost for each class. However, in practical situations, it is usually difficult to determine the real misclassification costs for different classes. Focusing on this problem, Tsung et al. designed a focal loss function through reconstructing the standard cross-entropy loss in which adjustment factors were added to make adjustments to unbalanced samples. This method achieved a good performance in object detection tasks [36]. Based on this, He et al. proposed the spatial-temporal multiscale neural network (STMNN) and trained the model with focal losses, which effectively solved the unbalanced issue [37]. Although the abovementioned algorithm-level methods have achieved good results, these methods mostly instruct the network to adjust the unbalanced data during training and ignore the importance of the feature-extraction process.

It has been demonstrated by some research works [38–41] that transfer learning and information fusion both play very important roles in feature extraction. For transfer learning, it may be viable to transfer the features of balanced data to unbalanced data, thereby diminishing the negative impacts of the unbalanced issue. For information fusion, the amount of information acquired by the network from the features can be increased by fusion [42], thereby upgrading the network's confidence. Motivated by the abovementioned methods, this paper focuses on both feature-extraction methods and algorithm-level learning strategies, and presents an invariant temporal-spatial attention fusion network (ITSA-FN) to solve the unbalanced data issue. The contributions are summarized as follows:

1. Proposed method designs an invariant temporal-spatial attention fusion network for feature extraction and inference representation of unbalanced data, which has achieved sound results.
2. A new joint constrained focal loss is designed, which is capable of facilitating the network's learning of relevant features from the algorithm aspect and adjusting the negative impacts of unbalanced data.
3. This article designs comparative experiments, ablation studies, and generalization performance analysis on vibration and current datasets with a variety of unbalanced ratios, and validated the effectiveness and superiority of our proposed model.

The rest of the paper is organized as follows.  Section 2 introduces the theoretical background, while Section 3 describes in detail the framework and learning strategy of our proposed method.  Section 4 discusses the experiments, including the experimental datasets, experimental details, network parameters, and experimental result analysis.  Section 5 presents the conclusions of this study and suggests future research directions.

## 2. Theoretical Background

In this section, we provide introductions to the theory of the network models, convolutional auto-encoder (CAE), and convolutional block attention module (CBAM) used in this paper.

### 2.1. CAE

A CAE is a combination of a convolutional neural network (CNN) and an auto-encoder (AE), which is a more efficient unsupervised feature extractor. Compared with an AE, a CAE replaces the fully connected layer with a convolutional layer and a pooling layer (downsampling layer) in the encoder and utilizes a deconvolution layer and an upsampling layer in the decoder. The computation process is as follows.

During encoding, let the input samples be *x*_m_. After the convolution and pooling operations, the feature maps of the hidden layer can be written as [43]

(1) $$\begin{array}{c} h\left(x_{m}\right)=\text{pool}\left(\sigma_{1}\left(x_{m}*W^{k}+{\text{b}}^{\text{k}}\right)\right), \end{array}$$

where “W” contains the initialized convolution kernels, the total number of which is *k*; “b” denotes a bias of convolutional kernel; “*σ*_1_” is the activation function; “^*∗*^” denotes the convolution operation; and “pool” denotes the pooling operation. The convolution of the kernels and the input *x*_m_ generates *k* feature maps *h*(*x*_m_).

During decoding, an unreasonable kernel size may lead to matrix block overlapping during deconvolution. Therefore, this paper replaces the deconvolution step with upsampling and convolution, and recovers the input size through nearest-neighbor interpolation during upsampling. However, since upsampling has already recovered the feature map size, it is sufficient to conduct a simple convolution, as illustrated in the following [43]:

(2) $$\begin{array}{c} \mathrm{R=}\sigma_{1}\left(r*{\hat{W}}^{k}+{\hat{b}}^{k}\right), \end{array}$$

where “*σ*_1_” is the leaky ReLU activation function, “$\hat{W}$” is the convolution kernel of the decoder, “$\hat{b}$” is the bias of the decoder, “r” is the hidden layer feature map *h*(*x*_m_) after size recovering through upsampling interpolation, and “R” consists of the reconstructed data.

### 2.2. Convolutional Block Attention Module

CBAM is a simple yet effective feed-forward neural-network attention module. As illustrated in Figure 1, for a given intermediate feature mapping F ∈ *ℝ*^*C*×*H*×*W*^ as input, the module infers the attention mappings along two independent dimensions (channel and spatial) in order. The computational equations can be written as [44]

(3) $$\begin{array}{c} {\text{F}}^{\prime }=M_{c}\left(F\right)=\sigma_{2}\left(\mathrm{MLP}\left(\text{AvgPool}\left(F\right)\right)+\mathrm{MLP}\left(\text{MaxPool}\left(F\right)\right)\right),\\ {\text{F}}^{\prime \prime }=M_{s}\left({\text{F}}^{\prime }\right)=\sigma_{2}\left(f^{7\times 7}\left(\left[\text{AvgPool}\left({\text{F}}^{\prime }\right);\text{MaxPool}\left({\text{F}}^{\prime }\right)\right]\right)\right), \end{array}$$

where “⊗” denotes elemental multiplication, “CBAM” is the convolutional block attention module, “F′” is output of channel attention mapping, “F″” is output of channel-spatial attention mapping, *M*_c_ ∈ R^C×1×1^ is the 1D channel attention mapping, *M*_s_ ∈ *R*^1×H×W^ is the 2D spatial attention mapping, “MLP” is the multilayer perceptron mapping representation, “AvgPool” is the average pooling operation, and “MaxPool” is the maximum pooling operation.

*f* ^7×7^ denotes convolution with filters of size 7 × 7. “*σ*_2_” is the sigmoid activation function.

## 3. The Proposed Method

Targeting the issue of unbalanced fault categories in actual situations, as illustrated in Figure 2, this paper presents an ITSA-FN model, which combines pretrained CAE modules, CBAM block, and LSTM for temporal-spatial feature extraction, and uses MLP to fuse and infer different modal features. Otherwise, we train the model with a newly designed joint normalized constrained loss function.

### 3.1. Invariant Temporal-Spatial Attention Fusion Neural Network

#### 3.1.1. Transfer Feature Extraction

To relieve the biased learning issue (e.g., where the network leans toward classes with larger sample populations) of the feature-extraction network (i.e., CAE) due to unbalanced samples, this paper adopts a transfer-learning method. First, this article trains the feature CAE with balanced samples under ideal experimental conditions. Then, after learning the distributions of the balanced samples, the unbalanced vibration signal (*x*_v_) and current signal (*x*_c_) are fed into the network for fine-tuning, thereby obtaining the data's low-level features. This is the encoding-decoding process, which can be expressed as follows:

(4) $$\begin{array}{c} h_{m}\left(x_{m}\right)=CAE_{m}^{\text{encoder}}\left(x_{m};\theta_{m}^{\text{encoder}}\right),m\in \left\{v,c\right\},\\ R_{m}=CAE_{m}^{\text{decoder}}\left(h_{m}\left(x_{m}\right);\theta_{m}^{\text{decoder}}\right),m\in \left\{v,c\right\}, \end{array}$$

where *h*_m_(*x*_m_), *R*_m_, *θ*_m_^encoder^, *θ*_m_^decoder^, CAE_m_^encoder^, and CAE_m_^decoder^ denote the pretrain CAE encoding representation, decoding (reconstruction) representation, encoder network parameter, decoder network parameter, encoder network section, and decoder network section of modal m, respectively. In addition, the structure of the pretrained model is illustrated in Figure 3, in which the module in green is the reserved model, and the section in gray is the classifier that guides the network during supervised training.

#### 3.1.2. Temporal-Spatial Attention Feature Representation

It has been proved by some research [45–47] that fault signal sequences are spatially and temporally correlated, and fault symptoms concentrate in the vicinity of the triggering time. Applying an attention mechanism and adopting a network with memory functionalities can make the network focus actively on the vicinity around fault moments and capture the contextual information, respectively, thereby improving the learning efficiency of fault features [48, 49]. Therefore, in this paper, we adopt the CBAM module, which is capable of capturing channel attention and spatial attention, and the LSTM to acquire the spatial-temporal characteristics of the faults and facilitate the network's ability to concentrate on learning fault information. The process is as follows.

First, CBAM is applied to the obtained encoding representations of the two modalities to obtain the spatial characteristics, which can be written as

(5) $$\begin{array}{c} Att_{m}=CBAM_{m}\left(h_{m}\left(x_{m}\right);\theta_{m}^{CBAM}\right),m\in \left\{v,c\right\}, \end{array}$$

where Att_m_, CBAM_m_, and *θ*_m_^CBAM^ denote the attention representation, the convolutional block attention network, and the attention network parameter of modal m, respectively.

Then, the attention representation is fed into the LSTM network to acquire the temporal characteristics, which can be written as

(6) $$\begin{array}{c} {\text{M}}_{m}=LSTM_{m}\left(\mathrm{At}t_{m};\theta_{m}^{LSTM}\right),m\in \left\{v,c\right\}, \end{array}$$

where *M*_m_, LSTM_m_, and *θ*_m_^LSTM^ denote the spatial-temporal attention representation, the LSTM network, and network parameter of modal m, respectively.

#### 3.1.3. Fusion Inference Representation

Information-fusion methods can improve the network's confidence by increasing the information volume. Therefore, from the point of view of information fusion, this paper fuses the data of two modalities (vibration and current) to optimize network performance, and the process is as follows.

After acquiring the spatial-temporal attention representation of the two modalities, we concatenate and fuse them into fusion representation

(7) $$\begin{array}{c} \text{Fusion}=M_{v}⊕M_{c}, \end{array}$$

where “⊕” denotes vector concatenation, and “Fusion” denotes the fusion vector after concatenation. Then, the fusion spatial-temporal attention representation is fed into the inference network (MLP) for fusing and fault inferences, which can be written as

(8) $$\begin{array}{c} Inf=MLP\left(\text{Fusion};\theta^{MLP}\right), \end{array}$$

where “Inf” denotes the inference output, “*θ*^MLP^” is the inference network parameter, and “MLP” is the multilayer perceptron with leaky ReLU and tanh activation functions.

### 3.2. Learning Strategy

This article designs a new normalized constrained loss function based on the imbalanced issue and the network structure, which will be described in detail in this section.

#### 3.2.1. Task Loss

The focal loss can self-adaptively adjust the impacts from a variety of sample populations through the addition of adjustment factors to the cross-entropy loss. Therefore, in order to better solve the issue of unbalanced sample, this paper adopts the focal loss as the task loss to guide network's learning, the computation equation of which can be written as [36]

(9) $$\begin{array}{c} L_{\text{focal}}\left(P\right)=-\alpha {\left(1-P\right)}^{\gamma }\text{log}\left(P\right), \end{array}$$

where “P” denotes the probability of a sample's correct classification, “*α*” denotes a weighting factor, and (1 − *P*) *γ* denotes the adjustment factor, where “*γ*” is the adjustable focal parameter. In addition, P = Inf is the inference network output (*α* = 0.25, and *γ* = 2).

#### 3.2.2. Recon Loss

The recon loss aims to minimize the distance between the input data and the reconstructed data. It is used in the fine-tuning training of a pretrained CAE model. In addition, integrating the recon loss into learning can facilitate the network's learning of trivial representations and suppress input noise. This paper utilizes the mean squared error as the recon loss, the computation equation of which can be written as [50]

(10) $$\begin{array}{c} L_{m}^{\mathrm{recon}}={\left\|x_{m}-R_{m}\right\|}_{2}^{2},m\in \left\{\mathrm{v,c}\right\}, \end{array}$$

where *x*_m_ and *R*_m_ denote the original input data and the reconstructed data, respectively, and ||·||_*2*_^*2*^ denotes the square of the *L*_2_ norm.

#### 3.2.3. Similarity Loss

When performing the fusion task, directly inputting the connected feature of each modality into the MLP fusion layer will make the network unable to effectively explore the interactions between the modalities, resulting in the problem of uncomprehensive fusion representation. Therefore, to obtain more comprehensive fusion representations, this paper adds a similarity constraint between the spatial-temporal attention representations of the two modalities to facilitate the network's capturing of invariant spatial-temporal attention representations. The central moment deviation (CMD) metric measures the distance between two distributions through matching differences between high-order moments. Its computation is simple and efficient, and capable of reducing the computation cost of the network [51]. Therefore, this article utilizes CMD as the similarity loss, the definition of which can be written as follows.

Let *X* and Y be bounded random samples having distributions of *p* and *q* in the tight interval of [a, b]^N^, respectively. Then, the central moment deviation normalizer CMD_K_ can be defined as empirical estimation of CMD metric as follows [51]:

(11) $$\begin{array}{c} CMD_{K}\left(X,Y\right)=\frac{1}{b-a}{\left\|E\left(X\right)-E\left(Y\right)\right\|}_{2}+\sum_{k=2}^{K}{\left\|C_{k}\left(X\right)-C_{k}\left(Y\right)\right\|}_{2}, \end{array}$$

where Ck and E(X) can be written as follows:

(12) $$\begin{array}{c} C_{k}\left(X\right)=E\left({\left(x-E\left(X\right)\right)}^{k}\right)E\left(X\right)\\ =\frac{1}{\left|X\right|}\sum_{x\in X}x, \end{array}$$

where E(X) is the empirical expectation vector of sample X, and Ck(X) is a vector on the *x*-axis of the central moment of all samples of order *k*. The CMD similarity loss used in this paper can be written as follows:

(13) $$\begin{array}{c} L_{sim}=CMD_{K}\left(M_{v},M_{c}\right). \end{array}$$

#### 3.2.4. Triplet Loss

Before the fusion of invariant spatial-temporal attention representations, to ensure high-level similarity relationships between the two modalities, this paper minimizes the distance among all samples with a similar semantic (class) from different modalities through the addition of a triplet boundary constraint Ltrip while maximizing the distance among representations without similarities [52]. For the vibration modal, we construct a triplet representation of (*M*v, M*c*+, and M*c*−) in which the current representation is semantically positively correlated with vibration representation *M*v, while the current representation M*c*− is negatively correlated with *M*v. Then, the triplet boundary loss with the vibration modal as the anchor can be written as [52]

(14) $$\begin{array}{c} L_{trip}^{v}=\text{max}\left(d\left(M_{v},M_{c}^{+}\right)-d\left(M_{v},M_{c}^{-}\right)+\text{margin},0\right). \end{array}$$

Similarly, the triplet boundary loss with the current modal as the anchor can be written as follows:

(15) $$\begin{array}{c} L_{\text{trip}}^{c}=\text{max}\left(d\left(M_{c},M_{v}^{+}\right)-d\left(M_{c},M_{v}^{-}\right)+\text{margin},0\right), \end{array}$$

where “d” denotes the Euclidian distance ||·||_2_^2^, “margin = 1” denotes the boundary value (ensuring that the loss function *L*_trip_ ≥0), and *M*_c/v_ denotes the invariant spatial-temporal attention representations of the two modalities.

Combining (14) and (15), this paper obtains the overall triplet boundary loss as follows:

(16) $$\begin{array}{c} L_{\text{trip}}=L_{trip}^{v}+L_{trip}^{c}. \end{array}$$

#### 3.2.5. Total Loss

In summary, this paper combines the abovementioned losses and proposes a new joint constrained focal loss function as follows:

(17) $$\begin{array}{c} L_{\text{total}}=L_{\text{focal}}+\beta L_{v}^{\text{recon}}+\lambda L_{c}^{\text{recon}}+\eta L_{\text{sim}}+\delta L_{\text{trip}}, \end{array}$$

where *β*, *λ*, *η*, and *δ* denote the adjustment factors of the loss function that adjust the contributions from each loss. This paper trains the network by minimizing this objective loss. The experimental procedures and details will be described in Section 3.3.

### 3.3. Methodology Procedures

In this section, we introduce the procedures of the method. The flowchart is shown in Figure 4.

According to the content in Figure 4, the details of the method steps are as follows:

1. Step 1: Preprocess the data. Experiment normalizes the vibration and current input data into the interval [−1, 1] and converts the normalized 1D data segments into 2D through reshaping, so that they could be fed into the 2D convolutional layer (i.e., the data are reshaped from 400 × 400 into 400 × 1 × 20 × 20).
2. Step 2: Acquire the pretrained CAE model. Experiment inputs the preprocessed source domain data (vibration and current) into our designed CAE network and then conducts the training and saves the resultant optimal model.
3. Step 3: Acquire the low-level feature representations. Experiment inputs the preprocessed target domain data into the pretrained model obtained in Step (2) and acquires the encoding and decoding representations of the CAE to guide the network in further learning.
4. Step 4: Acquire the spatial-temporal attention feature representation. Experiment inputs the encoding representation obtained in Step (3) into the CBAM module and LSTM network in order, thereby obtaining the spatial-temporal attention representations of the two modalities.
5. Step 5: Acquire the fusion inference representations. Experiment concatenates the spatial-temporal attention feature representations of the vibration and current datasets obtained in Step (4) and inputs them into the MLP for fusion, thereby obtaining the final inference representation.
6. Step 6: Compute the loss function. Experiment calculates the loss function for each component, respectively, according to the learning strategy and calculates the total objective loss L_total_ with the adjustment factors.
7. Step 7: Iteration and training. Experiment minimizes the total objective loss to train proposed network.
8. Step 8: Save the optimal model. Experiment saves the resultant optimal model for testing.

## 4. Experiment Results and Discussion

This section mainly discusses the experimental datasets, the network configuration, and the experimental procedures.

### 4.1. Datasets

To validate the effectiveness of proposed approach, this paper conducts experiments on bearing damage datasets released by the University of Paderborn, Germany [53]. The datasets consist of manual damages and accelerated lifetime damages in two sections. To be closer to practical situations, this paper adopts the accelerated lifetime damage data.

Specifically, the data experiments used are as follows. This paper considers two different operating conditions: the target domain (rotational speed *N* = 900 rpm, load torque *T* = 0.7 Nm, and radial force *F* = 1000 N) and the source domain (rotational speed *N* = 1500 rpm, load torque *T* = 0.1 Nm, and radial force *F* = 1000 N). The measured vibration and current signals of the equipment assembled with bearings under five different health statuses are illustrated in Table 1, in which each operating condition (rotational speed, torque, and radial force) contains data files collected by 20 sensors. This article selects one from them for experiment. Furthermore, this paper extracts 160,000 (400 × 400) data points from each file for experiments (in which one sample has 400 data points; thus, there were a total of 400 samples) and partitions them with a ratio of 3 : 1 into the training set and testing set, respectively.

Furthermore, we configure the distribution of our experimental data in the manner illustrated in Table 2, which lists the sample population of each class under different unbalanced ratios.

### 4.2. Experimental Network Configuration

This paper conducts the experiments with the open-source machine-learning framework PyTorch. The environment configurations are shown as follows: (1) CPU (AMD Ryzen 5 2600X Six-Core Processor, 3.60 GHz), (2) 16 GB of RAM, (3) GPU (NVIDIA GeForce GTX 1660, 6G), and a (4) code library and environment (PyTorch = 1.2.0 and Python = 3.7.9, respectively).

In addition, this paper selects network hyperparameters using a grid search algorithm, in which the optimal parameters are selected from the following finite sets: *β* ∈ {0.6, 0.7, 0.8, 0.9, 1.0}, *λ* ∈ {0.1, 0.2, 0.3, 0.4, 0.5}, *η* ∈ {0.5, 0.6, 0.7, 0.8, 0.9, 1.0}, *δ* ∈ {0.01, 0.1, 0.2, 0.3}, K ∈ {1, 2, 3, 4, 5}, lstm dim ∈ {32, 50, 64}, and mlp dim ∈ {128, 256, 512, 1024}, where *β*, *λ*, *η*, and *δ* are the adjustment factors of the loss function; K is the CMD order; “lstm dim” is the LSTM hidden layer dimension; and “mlp dim” is the MLP dimension. The grid searching saves the optimal model and returns the respective hyperparameters, as illustrated in Table 3.

This article configures the optimizer, learning rate, random seed, epoch, and batch size to be “Adam,” 0.01, 123, 300, and 100, respectively, for the training. In addition to these key hyperparameters, the structural details of our network components are illustrated in Figure 5.

### 4.3. Results and Discussion

For an effective validation of the proposed method, in this subsection, this paper designs comparative experiments, ablation studies, and generalization performance experiments.

#### 4.3.1. Experiment Analysis

In this subsection, for unbalanced samples (vibration and current) of different class population ratios, this paper designs a single modal (vibration or current) fault diagnosis model based on a CNN, CAE, a CNN with long short-term memory (CNN + LSTM), and two modal fusion models based on convolutional fusion neural network (CNN-fusion) and CAE fusion neural network (CAE-fusion) to compare with our proposed model. The structure of comparative model is illustrated in Figure 6, where the parameters of the convolutional layer and the MLP are identical to our network. The comparative experiments results are listed in Tables 4 and 5.

It can be observed from the results of the single modal methods that the vibration signal features are more prominent than those of the current signal, which is consistent with practical situations. Compared with CNN, the CNN-LSTM model achieves better performance under the different unbalanced conditions, and this benefits from the memory functionality of LSTM. In addition, compared with the single modal methods, it can be clearly observed that the fusion models show obvious improvements in diagnosis performance. This means that the network's confidence and performance can be effectively upgraded from the richer information obtained through the fusion feature.

In order to further validate the superiority of our network's classification performance, we visualize the confusion matrices of CNN-LSTM (vibration modal), CNN-fusion, CAE-fusion, and our method in Figure 7 with an unbalanced ratio of 10 : 5 : 4 : 3 : 2. It can be observed from the confusion matrices that our approach achieves the best classification performance in each fault category. This may be because our model integrates the spatial-temporal characteristics in the feature representations and adopts a reasonable constrained-learning strategy. Therefore, in order to validate the performance and rationality of our method, we carry out further analysis below.

#### 4.3.2. Visualization Analysis

In this subsection, we validate the rationality and effectiveness of our method through T-distributed stochastic neighbor embedding (T-SNE) from an intuitive perspective.

To reduce the workloads, this paper carries out the experiments with a representative unbalanced dataset (with an unbalanced ratio of 10 : 5 : 4 : 3 : 2) and performs a T-SNE visualization analysis on our network's feature representation process. As illustrated in Figure 8, the five plots show the distributions of the semantic features of the original input, encoder representation, spatial-temporal attention representation, MLP fusion representation, and the final inference representation. In each plot, the dots in different colors represent samples of different classes. In addition, the closer the dots of the same color and the farther away from the dots of different colors, the better the network's performance. It can be observed from Figure 8 that the samples' clustering effect becomes better in the order of network's modules. This means that the process of our network is reasonable when it carries out a fault diagnosis under unbalanced conditions.

#### 4.3.3. Ablation Studies Analysis

In the previous subsection, this paper visualizes the representation process of our network and validated the network's classification performance through the confusion matrices. However, there is a lack of quantitative assessment indices that could assess the model's performance. Therefore, in this subsection, this paper conducts an ablation study on the model's structural design and learning strategy, and utilizes the inference accuracy as an assessment index (unbalanced ratio = 10 : 5 : 4 : 3 : 2). The results are illustrated in Table 6.

It can be observed from the loss function results in Table 6 that the network is most sensitive to the focal loss. Because when it is used as the task loss, it has decisive impacts on the network's output, and its penalty mechanism can effectively suppress the influences of unbalancing. The similarity loss also has a relatively large impact on our network, due to that acquiring the invariance between the two modalities using this loss function before fusion can reduce the computation load while obtaining more comprehensive fault features. The recon loss has a relatively small impact on the network because the task loss can learn the trivial representations without this loss function. The impact of the triple loss is the smallest, since both the fusion and the similarity loss can achieve the clustering of this loss function, thereby weakening its contribution. Furthermore, it can be observed from the ablation experiment results of the network structure that each module (pretrain CAE, MLP, LSTM, and CBAM) has a positive impact on the network. This indicates that the design of proposed network is reasonable and effective.

#### 4.3.4. Generalization Performance Analysis

To validate the generalization capability of our model, in addition to the bearing data from the University of Paderborn, this paper used bearing-data from Xi'an Jiaotong University (XJTU-SY) and Case Western Reserve University (CWRU) for testing.

The data from the University of Paderborn consist of vibration signals from two sensors in the target domain dataset of the experiment section. The data from XJTU-SY include vibration signals of five fault categories for the outer ring, inner ring, outer ring + inner ring, bearing cage, and inner ring + ball + cage. The data from CWRU contain vibration signals from five categories of ball fault (fault diameter = 0.007 inches), ball-1 fault (0.014 inches), inner ring fault (0.007 inches), outer ring fault (0.007 inches), and normal condition. The test results are illustrated in Figure 9. It can be observed that our proposed model can still achieve good performance on the different datasets under a variety of unbalanced conditions, which has proved that our model has sound generalizing capability.

## 5. Conclusions

Focusing on the issue of unbalanced bearing fault samples, we found that in addition to resampling methods and algorithm-level strategies, transfer learning and feature fusion methods can effectively improve the network's reasoning performance under unbalanced conditions. Moreover, we also discover that obtaining modal invariance through similarity measurement constraints can improve the efficiency of feature fusion, thereby further improving network performance. Therefore, this paper innovatively combines the algorithm-level strategy (focal loss), transfer learning, and the feature fusion method under similarity constraints, and presents an ISTA-FN model for vibration and current signals. The model consists of two sections of invariant spatial-temporal representation and constrained fusion representation. The invariant temporal-spatial attention representation section includes a pretrained CAE model (trained by balanced samples), CBAM, and LSTM. The fusion representation section includes an MLP. First, we extract independent features and modal-invariant features (interactive features) of the vibration and current signals using the invariant temporal-spatial attention representation section. Then, we use MLP to fuse and infer the features of the two modalities and guide the network's learning through a new loss function. Finally, this paper validates the effectiveness of our model through experiments and a visualization analysis. However, our approach has not touched on the situation of an extremely small sample population which we plan to investigate in future research using a zero-sample learning method.

## Figures and Tables

**Figure 1:** The framework of CBAM.

**Figure 2:** The framework of ITSA-FN.

**Figure 3:** The framework of pretrain CAE.

**Figure 4:** The flowchart of the method.

**Figure 5:** The structure setting of ITSA-FN.

**Figure 6:** The structure of comparative model.

**Figure 7:** The confusion matrices.

**Figure 8:** T-SNE visualization.

**Figure 9:** Generalization experiment of ITSA-FN.

**Table 1:** Dataset interpretation.

Data domain	Code	State	Element	Combination	Extent	Speed	Torque	Radial force
Target domain	K001	Normal	—	—	—	900	0.7	1000
	KA04	Pitting	Outer ring	Single	1	900	0.7	1000
	KA15	Identification	Outer ring	Single	1	900	0.7	1000
	KB27	Pitting	Outer/inner ring	Multiple	2	900	0.7	1000
	KI21	Pitting	Inner ring	Single	1	900	0.7	1000

Source domain	K001	Normal	—	—	—	1500	0.1	1000
	KA04	Pitting	Outer ring	Single	1	1500	0.1	1000
	KA15	Identification	Outer ring	Single	1	1500	0.1	1000
	KB27	Pitting	Outer/inner ring	Multiple	2	1500	0.1	1000
	KI21	Pitting	Inner ring	Single	1	1500	0.1	1000

**Table 2:** Unbalanced data distribution.

Imbalance rate\code	K001	KA04	KA15	KB27	KI21
10 : 5	400	200	200	200	200
10 : 4	400	160	160	160	160
10 : 3	400	120	120	120	120
10 : 2	400	80	80	80	80
10 : 1	400	40	40	40	40
10 : 1 : 5 : 5 : 5	400	40	200	200	200
10 : 5 : 1 : 5 : 5	400	200	40	200	200
10 : 5 : 5 : 1 : 5	400	200	200	40	200
10 : 5 : 5 : 5 : 1	400	200	200	200	40
10 : 5 : 4 : 3 : 2	400	200	160	120	80

**Table 3:** Hyperparameter settings.

Hyperparameter	Value
*β*	0.7
*λ*	0.1
*η*	1.0
*δ*	0.1
*K*	3
lstm dim	64
mlp dim	128

**Table 4:** Experimental results I.

Method\ratio	10 : 5	10 : 4	10 : 3	10 : 2	10 : 1
CNN	93/76.33	92.69/73.85	90.91/70.91	89.44/68.88	87.14/71.43
CAE	92.33/78.33	90.77/70.38	92.73/73.64	91.67/71.11	89.29/67.14
CNN-LSTM	93.33/76	92.31/76.54	91.82/72.73	90.55/70	88.57/71.43
CNN-fusion	94.33	95	93.64	93.33	91.43
CAE-fusion	94	93.46	94.09	93.89	92.14
Our method	96.33	96.92	96.81	96.67	95

Index: accuracy: unit: %: Note: the first three are the test results of the single-mode method (the left is vibration, and the right is current).

**Table 5:** Experimental results II.

Method\ratio	10 : 1 : 5 : 5 : 5	10 : 5 : 1 : 5 : 5	10 : 5 : 5 : 1 : 5	10 : 5 : 5 : 5 : 1	10 : 5 : 4 : 3 : 2
CNN	92.31/70.77	91.54/70.38	91.54/72.69	91.92/73.46	91.66/73.33
CAE	92.69/71.92	88.85/71.15	89.61/70.38	89.23/75	87.5/75.42
CNN-LSTM	94.61/72.31	91.92/74.23	93.08/73.46	92.69/75.77	92.92/74.17
CNN-fusion	95.38	94.23	93.85	94.23	94.17
CAE-fusion	95.77	93.46	94.23	94.61	94.16
Our method	97.69	96.15	96.54	97.69	97.08

Index: accuracy: unit: %: Note: the first three are the test results of the single-mode method (the left is vibration, and the right is current).

**Table 6:** Experiment of ablation studies.

Experiment type	Ablation factors	Accuracy (%)
Loss ablation	Without focal loss	93.33
	Without recon loss	95.42
	Without similarity loss	94.58
	Without triplet loss	96.67
Structure ablation	Without CBAM	95.83
	Without LSTM	94.58
	Without MLP	94.17
	Without pretrain CAE	95
—	None	97.08

## Data Availability

The Paderborn bearing dataset was used in our study, which is publicly available via the following link: https://mb.uni-paderborn.de/kat/forschung/datacenter/bearing-datacenter/. The CWRU bearing dataset was used in our study, which is publicly available via the following link: https://engineering.case.edu/bearingdatacenter. The XJTU-SY bearing dataset was used in our study, which is publicly available via the following link: https://biaowang.tech/xjtu-sy-bearing-datasets/.
